This article has been retracted.

# Analysis of the Model for Sports Enhancing Human Health Using Data Mining

**DOI:** 10.1155/2022/3416255

**Published:** 2022-02-11

**Authors:** Ruiqing Wang, Lei Han

**Affiliations:** ^1^School of Physical Education, Harbin University, Harbin 150086, China; ^2^School of Environmental and Chemical Engineering, Dalian Jiaotong University, Dalian 116028, China

## Abstract

The problems of low reliability and the high fitting degree of mutual information feature extraction of traditional sports to human health enhancement model are analyzed. We analyze and study the sports to human health enhancement model using data mining. The model consists of a data layer, a logic layer, and a presentation layer. Sports project data, real-time sports data, and health monitoring data are collected in the data layer, and the collected data are transmitted to the logic layer. The logical layer uses the dynamic difference feature classification algorithm of data mining to fuse human health data, extract the mutual information features of human health, and input the features into the long short-term memory (LSTM) neural network, which outputs the pattern recognition results of sports health after forward and reverse operations. The results of sports health pattern recognition are input into the display layer, and the enhancing effect of sports on human health is presented for users by constructing a model of sports on human health. The results show that the effect of sports on human health enhancement analyzed by the model in this paper is extremely accurate, which can significantly improve the health level of community residents and college students. When the number of data is about 600, it remains at about 0.05, indicating that this model has high reliability, and the fitting degree of mutual information feature extraction is up to 99.82%. It has certain practical application value.

## 1. Introduction

Obese people have a higher incidence of hypertension, arteriosclerosis, and osteoporosis. Therefore, more and more people pay attention to their health. Kenneth Cooper, an American expert, put forward that as long as you participate in sports, you will benefit, and sports are additives to human health. As early as in the BC period, Aristotle also proposed the idea of “life lies in movements.” Many sports health concepts and living habits promote people to exercise more and more. However, different exercise intensities and exercise modes can enhance human health at varying degrees. At present, there is no reasonable evaluation system or model to evaluate such problems, so that people do not fully understand the relationship between exercise and health, and it is a long-term and continuous process for exercise to enhance human health, during which people cannot grasp the health enhancement effect of current kinds of exercise in time, which is easy to make the sports population lose their self-restraint on exercise. In the face of the above situation, Islam and Alajlan [1] designed a human health recognition model, analyzed the impact of sports on human health enhancement by analyzing the distance of aligning heartbeat within individuals and measuring the recognition ability of human health with different alignment methods, and obtained relevant analysis results. Baqueri et al. [2] established the exercise schedule of relevant research objects by simulating residents' travel and activities outside the study area, preprocessed all data with fees, and analyzed high-intensity tourism activities with relevant data to achieve the effect of human health enhancement. Parmezan Bonidia et al. [3] tested whether there were differences in exercise variability and complexity only above exercise intensity during running and whether exercise would increase running speed and neuromuscular fatigue. Combined with the analysis results and human physiological parameters, they constructed a model of sports enhancing human health and obtained relevant analysis results. Chen [4] studied the impact model of physical training on physical health. The model integrates sports training and diet management. Using the model, we can obtain such information as to whether people's current diet is reasonable and the impact of sports training intensity on their health. Zheng and Haifeng [5] studied the model of the effect of exercise with the same intensity on the amount of abdominal visceral fat, which can be used to obtain the changes of human visceral fat at different exercise intensities.

In the process of sports, the human body can produce a large amount of various data [6, 7], which makes the subsequent data analysis more difficult. Therefore, a model and analysis method of sports on human health enhancement is designed in this paper based on data mining. The main contributions of this paper are as follows: (1) Data mining is an algorithm that mines available information from a large amount of data. It is the most commonly used algorithm in machine learning algorithms. Using this algorithm can improve mining efficiency and accuracy. (2) The dynamic difference feature classification algorithm in data mining is used to fuse human health data, extract human health mutual information features, and input the feature into the LSTM neural network. The neural network outputs the results of motion health pattern recognition after forward and reverse operations, so as to improve the recognition accuracy. (3) The results of sports health pattern recognition are input into the display layer. Through constructing the model of sports on human health enhancement, the effect of sports on human health enhancement is presented to users, the visualization of relevant information is realized, and the impact results of their current sports behavior on their health enhancement are provided.

## 2. Methodology

### 2.1. Structure of Sports on Human Health Enhancement Model

According to the hierarchical concept, a model of sports on human health enhancement based on data mining is designed, as shown in Figure 1.

According to Figure 1, the human health enhancement model of sports based on data mining is composed of a data layer, a logic layer, and a display layer. The data layer is used to obtain the human body's sports project data, sports real-time data, and health monitoring data, and the above data are transmitted to the logic layer [8, 9]. The logic layer is used to extract the mutual information features of the human body's exercise data and health data. After sports health pattern recognition and logical calculation of sports intensity, the relevant calculation results are input into the display layer to provide users with sports project management, sports intensity viewing, sports health mode, and other information, so that users can fully understand the health enhancement effect of current sports.

### 2.2. Extraction of Features of Human Health Mutual Information

During exercise, the human body will produce a large number of health data, such as current pulse beat, blood circulation times, changes in body water, and fat [10, 11]. Their data sources are different, and their preservation formats are also different, forming a multisource heterogeneous complex data source. In order to extract useful health data from complex data sources, the dynamic difference feature classification method in data mining is used to fuse multisource heterogeneous human health data and extract human health mutual information features. The detailed process is as follows.

Let the scalar time series of human health data be *o*=[⋯,*o*_*i*_, ⋯,*o*_*j*_^*i*^, ⋯]^*T*^ ∈ *R*^*nN*^, and the dynamic difference feature classification method is used to decompose the scalar time series in the windowed time domain. The expression equation is as follows:

(1) $$\begin{array}{c} o\left(t\right)=\iint_{a,b}\rho \left(a,b\right)\frac{da\;db}{\sqrt{\left|a\right|}*a^{2}}\frac{f\left(t-b\right)}{f\left(t\right)}, \end{array}$$

where *f*(•) refers to transient sampling value at sampling time; *ρ*(*a*, *b*) refers to the joint distribution state of mutual information of human health data; *a* and *b* refer to matching parameters and frequency-domain decomposition spectrum; and *t* refers to the time.

Fuzzy control is applied to the time-domain sequence in the windowed area of equation (1) to mine the feature vector of human health data, and the state function expression equation of the feature vector is as follows:

(2) $$\begin{array}{c} o_{i}{}^{\prime }=\min\left\{f_{i}\left(o_{i},u_{i}\right)D\left(o_{i}\right)\right\}, \end{array}$$

where *o*_*i*_ refers to the vector of human health data distribution state, *u*_*i*_ refers to weight input vector, and *D*(*o*_*i*_) refers to eigenvector distribution distance.

The fuzzy clustering algorithm is used to cluster the time series mean of the results of equation (2) to obtain the linear average time series of human health data. The expression equation is as follows:

(3) $$\begin{array}{c} \langle o\left(n\right)\rangle =\frac{\sum_{n=1}^{N}x\left(o\right)}{N}, \end{array}$$

where *N* refers to the amount of human health data, and *n* ∈ *N*. The frequency response of the time series of linear average human health data is configured to obtain the autocorrelation feature state of human health data. The expression equation is as follows:

(4) $$\begin{array}{c} o_{n}=ot_{0}+no\Delta t=h\left(t_{0}+n\Delta t\right)+\omega_{n}, \end{array}$$

where *n* refers to the data dimension; *ω*_*n*_ refers to the phase space distribution interval when the dimension is *n*; *n*Δ*t* refers to the time interval; *t*_0_ refers to the initial time; and *h* refers to the rounding operation function.

The geometric invariants of human health data in phase space are calculated, and redundant interference data are removed [12]. The expression equation is as follows:

(5) $$\begin{array}{c} z\left(t\right)=s\left(t\right)+js\left(t\right)⊗h\left(t\right), \end{array}$$

where *j* refers to adjustable parameters; *j* refers to eigenvector amplitude; and *h*(*t*) refers to corrected periodic function.

After the redundant interference data of human health data are removed, the limited dataset of human health data is obtained by clustering algorithm [13]. The expression equation is as follows:

(6) $$\begin{array}{c} O=\left\{o_{1},o_{2},\cdots o_{n}\right\}\in R^{n}. \end{array}$$

Recursively process equation (6), perform differential evolution calculation on each data sample in the human health dataset, and obtain the output scalar timing of the human health dataset. The expression equation is as follows:

(7) $$\begin{array}{c} o={\left(o_{i1},o_{i2},\cdots ,o_{in}\right)}^{T}. \end{array}$$

Let the clustering category threshold be *ζ*. According to the threshold, the number of feature data clusters in the limited human health dataset is calculated. The expression equation is as follows:

(8) $$\begin{array}{c} V=\left\{v_{ij}\right\}, \end{array}$$

where *V*_*i*_ refers to the finite dataset clustering center of the *i* time-domain distribution feature point. The output component of data mining is calculated according to the clustering center. The expression equation is as follows:

(9) $$\begin{array}{c} \Delta o_{i}=a+bo_{n}-ao_{n}. \end{array}$$

The clustering center partition matrix of the data mining output component in equation (9) is calculated by using the perturbation variable difference algorithm. The expression equation is as follows:

(10) $$\begin{array}{c} U=\left\{\mu_{ik}\right\}. \end{array}$$

Equation (10) is normalized to obtain the mutual information features of human health data. The expression equation is as follows:

(11) $$\begin{array}{c} o_{i}{}^{\prime }=o_{i}/\left\|o_{i}\right\|. \end{array}$$

After the mutual information features of human health data are obtained according to the above equation, the LSTM neural network is used to identify the mutual information feature to obtain human sports health [14].

### 2.3. Human Sports Health Pattern Recognition

As we all know, human health models are divided into three models: healthy, subhealth, and unhealthy [15, 16]. In order to clearly show the effect of sports on enhancing human health after exercise, the three human health models are divided into three levels: I, II, and III. The smaller the level, the worse the health status in the health model. The mutual information features of human health data obtained in the previous section are input into the long-term and short-term memory neural network to identify human health patterns. The essence of human health pattern recognition is the classification and processing of signal sequences. Because human motion is a continuous process, the motions of the human body can be divided into several cycles [17, 18], and the human health pattern can be identified according to the time relationship of mutual information features of human health data. The process is as follows.

The internal state *c*_*t*_ is set in the LSTM neural network layer. Then, it is used to record the historical information before the deadline of a certain time, and the values of input gate, forgetting gate, and output gate of the LSTM neural network are calculated [19]. The expression equation is as follows:

(12) $$\begin{array}{c} \left\{\begin{array}{c} i_{t}=\sigma U_{i}h_{t-1}+\sigma \psi_{i}x_{t}+\sigma b_{i},\\ f_{t}=\sigma U_{f}h_{t-1}+\sigma \psi_{f}x_{t}+\sigma b_{f},\\ p_{t}=\sigma U_{0}h_{t-1}+\sigma \psi_{0}x_{t}+\sigma b_{0}, \end{array}\right. \end{array}$$

where *i*_*t*_, *f*_*t*_ and *p*_*t*_ are human health feature values output by input gate, forgetting gate, and output gate; *σ* refers to the activated function; *h*_*t*_ refers to the output value of the hidden layer of the neural network; *f*, *U*, and *ψ* refer to the nonlinear activation function, state weight matrix, and input weight matrix; and *b* refers to the offset value.

The numerical value of the internal state *c*_*t*_ of the LSTM neural network layer is calculated. The expression equation is as follows:

(13) $$\begin{array}{c} c_{t}=f_{t}*c_{t-1}+i_{t}*\;\tanh\;U_{c}h_{t-1}+i_{t}*\;\tanh\;\sigma_{c}x_{t}+i_{t}*\;\tanh\;b_{c}. \end{array}$$

The value *h*_*t*_ of the hidden layer output of neural network is calculated [20]. The expression equation is as follows:

(14) $$\begin{array}{c} h_{t}=p_{t}*\;\tanh\left(c_{t}\right). \end{array}$$

Equations (12) and (14) are the forward calculation of the LSTM neural network, but there are two hidden layers in the LSTM neural network [21]. In order to make the output human health model results more authoritative, the mutual information features of human health data are calculated again according to the forward calculation results [22].

Let *ϑ* be the forward calculation results of the LSTM neural network. The reverse calculation expression equation is as follows:

(15) $$\begin{array}{c} \left\{\begin{array}{c} \left[h_{t}^{f\_1},c_{t}^{f\_1}\right]=\vartheta \left(h_{t-1}^{f\_1},c_{t-1}^{f\_1},p_{t};\theta^{f\_1}\right),\\ \left[h_{t}^{f\_2},c_{t}^{f\_2}\right]=\vartheta \left(h_{t-1}^{f\_2},c_{t-1}^{f\_2},h_{t}^{f\_1};\theta^{f\_2}\right),\\ \left[h_{t}^{b\_1},c_{t}^{f\_2}\right]=\vartheta \left(h_{t-1}^{b\_1},c_{t-1}^{b\_1},p_{W+1-t};\theta^{b\_1}\right),\\ \left[h_{t}^{b\_2},c_{t}^{b\_2}\right]=\vartheta \left(h_{t-1}^{b\_2},c_{t-1}^{b\_2},h_{t}^{b\_1};\theta^{b\_2}\right), \end{array}\right. \end{array}$$

where *f*_1, *b*_1, *f*_2, and *b*_2 are the forward and reverse outputs of the first and second hidden layers of the LSTM neural network, respectively; *θ* refers to the weight parameters of hidden layer; and *o* refers to the output vector.

According to the above calculation method, the gradient Adam optimization algorithm is used to train the LSTM neural network model. The steps are as follows:

Step 1: use equations (12) to (14) to calculate the cell output value of the LSTM neural network.
Step 2: after inverse calculation with equation (15), the cross-entropy error term of the LSTM neural network is obtained. The expression equation is as follows:
  (16) $$\begin{array}{c} Loss_{i}=-\log\left(\left(e^{H*\psi_{0,i}}+b_{o,i}\right)/\overset{N}{\underset{j=1}{\sum }}e^{H*\psi_{o,j}}+b_{o,j}\right), \end{array}$$
where *H* refers to the output value of the hidden layer, *N* refers to the total number of human health mutual information features, and *Loss*_*i*_ refers to the classification loss of the LSTM neural network in recognizing human health patterns.
Step 3: according to the result of equation (16), the weight gradient of the human health mutual information feature is calculated.
Step 4: use the gradient Adam optimization algorithm to gradient the weight of human health mutual information features, and reinput the optimization results into the hidden layer of the LSTM neural network. After reverse calculation, the human health pattern recognition results are output, and the sports health pattern recognition results are input into the display layer. By constructing the model of sports on human health enhancement, the effect of sports on human health enhancement is presented to users.

The process of sports on the human health enhancement model is shown in Figure 2.

The data layer is used to collect sports data, real-time sports data, and health monitoring data, and the collected data is transmitted to the logic layer. The logic layer uses the dynamic difference feature classification algorithm in the data mining to fuse the human health data, extract the human health mutual information feature, and input the feature into LSTM neural network. The neural network outputs the results of sports health pattern recognition after forward and reverse operations. The results of sports health pattern recognition are input into the display layer, and the enhancement effect of sports on human health is presented to users by constructing the enhancement model of sports on human health.

## 3. Experimental Design and Result Analysis

### 3.1. Datasets and Experimental Indexes

The CPU of this experiment is Intel (R) Core (TM) i5-9400 and the operating system is Windows 10. The deep learning framework is the PyTorch deep learning framework. The development language is Python.

The 2019 sports health data of residents aged 30 to 40 years in a community and the sports health of college students in a university are taken as the experimental objects and labeled as dataset as A and dataset B, respectively. This model is used to recognize the physical health patterns of community residents and college students after exercise and analyze the effect of sports on human health. Dataset A: community residents use spacewalker, ladder, waist back massager, pedal, rib frame, Tai Chi massage device, leg pressing trainer, horse riding machine, and vertical waist twisting device for training and test the physiological parameters of residents every month. Dataset B: a university student participates in sports associations, such as basketball, badminton, volleyball, and other track and field sports, and tests the physiological parameters of residents every month. Dataset A and Dataset B are divided in such a way that 80% of the data are used for training and 20% of the data are used for testing.

In order to highlight the reliability of the model in this paper, experiments are carried out using the model in literature [1], literature [2], literature [3], literature [4], and literature [5]. The model in literature [1] to the model in literature [5] represent the heartbeat of the sport recognition model, outdoor sports model, high-intensity running linear analysis model, sports impact analysis model, and different intensity sports impact recognition model, respectively.

(1) Health enhancement effect of community residents and college students after sports: after the model in this paper is applied, the more the number of community residents and college students in a healthy state, the better the enhancement effect.
(2) Human health index of community residents and college students: the body mass index (BMI) is about 18, indicating that the healthier the community residents and college students are, the better the practical application effect of the model is.
(3) Human health pattern recognition accuracy: the model recognition results in this paper are compared with the actual health level. The closer the two values are, the higher the human health pattern recognition accuracy is. The calculation equation of this index is as follows:
  (17) $$\begin{array}{c} r=\frac{z}{x}\times 100\%, \end{array}$$
where *z* represents the amount of correctly identified human health model data and *x* represents the total amount of human health model data.
(4) Reliability test results: taking the classification loss value when identifying human health mode as the measurement index and dataset A as the experimental object, test the change of classification loss value during identification under different human health data samples. The loss value is calculated as follows:
  (18) $$\begin{array}{c} A=\frac{S}{K}, \end{array}$$
where *S* represents the amount of data lost in the classification process and *K* represents the total amount of data.
(5) Mutual information feature extraction fit: it refers to the similarity between feature extraction results and actual mutual information features.
  (19) $$\begin{array}{c} \mathrm{r=}\frac{z}{d}\mathrm{\times 100\%,} \end{array}$$
where *z* represents the number of mutual information features actually extracted and *d* represents the total amount of mutual information features.

### 3.2. Results and Discussion

#### 3.2.1. Comparison of Physical Health Enhancement Effect

In order to more clearly describe the practical application effect of this model, taking the proportion of different health models as the measurement index, this paper analyzes the health enhancement effect of community residents and college students after sports in 2019 as shown in Figure 3.

According to Figure 3, after using this model to output the human health enhancement data of community residents and college students after sports, it can be seen that the overall physical quality of community residents and college students has been enhanced. At the two time nodes at the beginning and end of 2019, the proportion of health in the health model of college students and community residents increased greatly, while the proportion of subhealth and unhealthy decreased. On the whole, the physical quality of college students is higher than that of community residents. The reason is that college students have regular work and rest time, diet, relatively young age, and rapid metabolism. On the contrary, the work and life pressure of community residents are relatively large, and different working hours or single dietary structure has a great impact on their health. In conclusion, this model can effectively identify human health patterns and has good applicability.

#### 3.2.2. Comparison of Changes in Human Health Index

Taking human health index BMI as the index and dataset A and dataset B as the experimental objects, this model is used to output the changes of BMI values of community residents and college students when they exercise for one year, as shown in Figure 4.

We observe from Figure 4 that the human health indexes of community residents and college students decrease with the increase of exercise months, and the human health index of college students is lower than that of community residents. The initial BMI of college students and community residents exceeded 20, but after continuous sports, their BMI decreased to about 18, which is the normal standard of the human body. The above results show that continuous sports can effectively improve the BMI of the human body and enhance physical quality.

#### 3.2.3. Comparison of Human Health Pattern Recognition Accuracy

Taking a resident in data set A as the experimental terrain and the recognition accuracy as the measurement index, this model is used to recognize the changes of the health model in 2019, compare it with the actual health model, and analyze the impact of sports on human health enhancement as shown in Figure 5.

It is seen from Figure 5 that the health grade output of the model in this paper is exactly the same as the actual health grade of the residents, and its output accuracy is as high as 100%. The resident kept doing sports in 2019, during which his health level gradually rose from the initial unhealthy level II to healthy level II. The above results show that the output results of this model are very accurate, and the output results can fully describe the enhancement effect of sports on human health and explain the change of residents' health level.

The accuracy of human health pattern recognition by different methods is detected, and the results are shown in Figure 6.

By analyzing the data in Figure 6, it can be seen that the accuracy of human health pattern recognition of the model in literature [1] varies from 79% to 88%, and the accuracy of human health pattern recognition of the model in literature [2] varies from 63% to 69%. The accuracy of human health pattern recognition of the model in literature [3] varies from 59% to 78%, and the accuracy of human health pattern recognition of the model in literature [4] varies from 63% to 76%. The accuracy of human health pattern recognition of the model in literature [5] varies from 52% to 58%. Compared with these methods, the accuracy of human health pattern recognition of this model is always more than 95%, which can realize the accurate recognition of human health patterns.

#### 3.2.4. Comparison of Reliability Test Results

The reliability test result is shown in Figure 7.

According to Figure 7, when analyzing the effect of sports on health enhancement, the loss value curves of the six models decrease rapidly with the increase of the amount of data before the amount of human health data is 1000, but when the amount of human health data exceeds 1000, the loss value curves of the six models are not affected by the amount of human health data, showing a gentle trend. The maximum loss value of this model is lower than that of the other five models, and it begins to show a stable trend when the amount of data is about 600, and the loss value is 0.05. The above results show that the loss value of this model in analyzing the effect of sports on human health enhancement is the smallest, and its output result is reliable.

#### 3.2.5. Comparison of Mutual Information Feature Extraction Fit

Taking 5000 groups of community residents' human health data in data set A as the experimental object, the fitness of mutual information features extracted by this model is tested, as shown in Table 1.

According to Table 1, the fit degree of the output results of the six models decreased with the increase of the health array. Before the health data group was 3000, the decrease of the fit of the output results of the six models was low. When the lecture data group continued to increase, the decrease of the fit of all model output results gradually increased. When the data group of the model in this paper is 5000 groups, the consistency of the output results is 98.01%, which is 3.91%, 8.09%, 7.94%, 7.9%, and 9.87% higher than the model in literature [1] and the model in literature [5]. From the above results, it can be concluded that the output results of the model in this paper have the highest fit, which shows that it has good applicability.

## 4. Conclusions and Future Works

This paper designs a model of sports to human health enhancement based on data mining and uses the model to analyze the sports health data of residents and college students in a community in 2019. The analysis results show that the physical quality of college students is slightly higher than that of community residents, but after continuous sports, their physical health BMI decreases to the standard value, indicating that continuous sports can effectively enhance human health. However, this study also has some shortcomings, that is, it does not use more data for experimental testing to verify the applicability of this model. Therefore, future work is to use more data to test the model based on this study to further verify the reliability of the experimental results.

## Figures and Tables

**Figure 1:** Structure of sports on the human health enhancement model.

**Figure 2:** The process of sports on the human health enhancement model.

**Figure 3:** Community residents and college students' physical health enhancement effect after sports. (a) Dataset A. (b) Dataset B.

**Figure 4:** Changes in the human health index of community residents and college students.

**Figure 5:** Comparison of human health pattern recognition results.

**Figure 6:** Comparison of human health pattern recognition accuracy.

**Figure 7:** Comparison of reliability test results.

**Table 1:** Comparison of mutual information feature extraction fit degree (%).

Human health data group	This model	Literature [1] model	Literature [2] model	Literature [3] model	Literature [4] model	Literature [5] model
500	99.82	99.81	97.64	99.24	98.57	95.46
1000	99.79	99.72	97.09	98.97	98.41	94.82
1500	99.75	99.70	96.88	98.54	98.24	93.55
2000	99.73	99.54	95.41	98.02	97.33	92.89
2500	99.68	99.46	95.03	97.55	96.06	91.77
3000	99.54	99.31	94.25	97.31	95.89	91.54
3500	99.33	98.09	94.06	95.88	95.13	90.49
4000	99.01	97.22	93.39	94.27	94.22	89.22
4500	98.86	96.55	92.17	93.05	93.09	89.03
5000	98.01	94.10	89.92	90.07	90.11	88.14

## Data Availability

The data used to support the findings of this study are available from the corresponding author upon request.
